RETRACTED

# Oxidized LDL Disrupts Metabolism and Inhibits Macrophage Survival by Activating a miR-9/Drp1/Mitochondrial Fission Signaling Pathway

**DOI:** 10.1155/2020/8848930

**Published:** 2020-11-01

**Authors:** Ting Xin, Chengzhi Lu, Jing Zhang, Jiaxin Wen, Shuangbin Yan, Chao Li, Feng Zhang, Jin Zhang

**Affiliations:** Department of Cardiology, Tianjin First Center Hospital, Tianjin, China

## Abstract

Mitochondrial dysfunction is associated with macrophage damage, but the role of mitochondrial fission in macrophage cholesterol metabolism is not fully understood. In this study, we explored the influences of miR-9 and mitochondrial fission on macrophage viability and cholesterol metabolism. Macrophages were incubated with oxidized low-density lipoprotein (ox-LDL) *in vitro*, after which mitochondrial fission, cell viability, and cholesterol metabolism were examined using qPCR, ELISAs, and immunofluorescence. ox-LDL treatment significantly increased Drp1-associated mitochondrial fission. Transfection of Drp1 siRNA significantly reduced cell death, attenuated oxidative stress, and inhibited inflammatory responses in ox-LDL-treated macrophages. Interestingly, inhibition of Drp1-related mitochondrial fission also improved cholesterol metabolism by balancing the transcription of cholesterol influx/efflux enzymes. We also found that miR-9 was downregulated in ox-LDL-treated macrophages, and administration of a miR-9 mimic decreased Drp1 transcription and mitochondrial fission, as well as its effects. These results indicate that signaling via the novel miR-9/Drp1/mitochondrial fission axis is a key determinant of macrophage viability and cholesterol metabolism.

## 1. Introduction

Atherosclerosis (AS) is a leading cause of ischemic heart disease. Among the molecular mechanisms underlying AS, inflammation response and lipid metabolism disorder have been identified as particularly important [1, 2]. At the molecular level, chronic hyperlipidemia induces endothelial dysfunction and thus promotes deposition of cholesterol on the vascular wall [3]. Smooth muscle cells and macrophages uptake excess cholesterol then migrate into the middle layer of vessel wall, contributing to the formation of plaques [4]. Therefore, increased intake and decreased efflux of cholesterol from macrophages have been identified as a key contributor to macrophage dysfunction, which is associated with the development of AS [5, 6]. However, cholesterol metabolism homeostasis in macrophages under hyperlipidemia stress conditions has not been well studied [7, 8].

Mitochondria serve as the primary energy source for cells by producing ATP through oxidative phosphorylation [9–12]. Properly functioning mitochondria consume glucose and cholesterol to generate ATP that supports macrophage metabolism. Predictably, mitochondrial dysfunction impairs cholesterol decomposition and leads to accumulation of cholesterol in macrophages, ultimately promoting formation of plaques [13, 14]. Mitochondria are therefore a potential target for therapies aiming to regulate cholesterol metabolism in macrophages [15, 16]. Many recent studies have reported that events that alter mitochondrial morphology, such as fission, fusion, and autophagy, have important effects on mitochondrial function [17–20]. Under normal conditions, mitochondrial fission increases the number of mitochondria in a cell and thus enhances mitochondria-dependent energy output [21]. Mitochondrial fusion enhances communication among mitochondria by allowing them to exchange DNA and metabolic substrates [22], which is vital for maintaining mitochondrial homeostasis. Mitochondrial autophagy, which is termed mitophagy [23], is a process by which damaged mitochondria are removed through lysosomes. Moderate mitophagy attenuates the number of dysfunctional mitochondria and promotes mitochondrial biogenesis [20, 24]. Together, these three mitochondrial morphology alterations act as upstream mediators of mitochondrial function. However, whether abnormalities in mitochondrial morphology are associated with cholesterol metabolism disorders in macrophages remains unknown.

RETRACTED

Biogenesis of endogenous microRNAs begins with the synthesis of primary microRNAs, or pri-miRNAs, in the nucleus [25]. pri-miRNAs are cut into hairpin RNAs called pre-miRNAs. pre-miRNAs are further cut into shorter double-stranded micro-RNAs, and RNA helicase then generates one or two mature single-stranded microRNAs [26]. MicroRNAs regulate gene expression by silencing translation of messenger mRNAs [26]. Mature single-stranded microRNAs bind to members of the Argonaute protein family to form an RNA-induced silencing complex (RISC) [27]. The target mRNA then binds to complementary bases in the 3′ noncoding region of the RISC [28]. The resulting destabilization or cleavage of the sigma region ultimately suppresses translation of the target mRNA. Recent studies have shown that microRNA can directly bind to an A/U- (adenine/uracil-) rich conserved element in the 3′ noncoding region of mRNA after the cell cycle stops to activate mRNA translation [29]. Through these mechanisms, microRNAs can regulate various cellular processes, including metabolism, division, differentiation, apoptosis, and autophagy [30]. Our previous studies demonstrated that macrophage functions and inflammatory response are regulated by miR-9. In addition, recent research has identified new roles for miR-9 in regulating mitochondrial function [31]. In this study, we explored the influence of miR-9 on macrophage viability and cholesterol metabolism with a focus on mitochondrial fission.

RETRACTED

## 2. Results

### 2.1. ox-LDL Activates Mitochondrial Fission and Inhibits Mitochondrial Fusion in Macrophages

To understand changes in mitochondrial dynamics in response to ox-LDL treatment, an immunofluorescence assay was used to examine mitochondrial morphology. As shown in Figures 1(a)–1(c), normal mitochondria were rod shaped and evenly dispersed throughout the cytoplasm of macrophages. After exposure to ox-LDL, numbers of fragmented mitochondria increased, indicating disturbances in mitochondrial dynamics. RNA analysis demonstrated that the Mff, Fis1, and Drp1 genes, which are related to mitochondrial fission, were significantly upregulated in response to ox-LDL (Figures 1(d)–1(i)). Interestingly, levels of the mitochondrial fusion-related genes Mfn2, Mfn1, and Opa1 decreased markedly after exposure to ox-LDL (Figures 1(d)–1(i)). Together, our data indicate that ox-LDL activates mitochondrial fission and inhibits mitochondrial fusion in macrophages.

### 2.2. Inhibition of Drp1-Related Mitochondrial Fission Attenuates ox-LDL-Induced Macrophage Death

To determine whether increased mitochondrial fission is required for ox-LDL-mediated macrophage damage, macrophages were transfected with siRNA against Drp1 and cell viability was then measured in a CCK-8 assay. As illustrated in Figure 2(a), compared to the control group, ox-LDL significantly decreased cell viability, and this effect was attenuated by Drp1 siRNA (siRNA/Drp1). The protective effect exerted by siRNA/Drp1 on macrophage viability was further examined in an LDH release assay. As shown in Figure 2(b), compared to the control group, ox-LDL promoted LDH release from macrophages into the medium. Loss of Drp1 through transfection of siRNA/Drp1 significantly reduced LDH release. Taken together, these results indicate that inhibition of Drp1 sustained macrophage viability. To further examine whether Drp1 knockdown was associated with increased cell viability, numbers of apoptotic cells were measured in a TUNEL assay. As shown in Figures 2(c) and 2(d), compared to the control group, numbers of TUNEL-positive cells increased after ox-LDL treatment. However, siRNA/Drp1 transfection inhibited ox-LDL-induced macrophage death, as evidenced by decreased TUNEL-positive cell numbers. Cell viability was also examined by analyzing the expression of caspase-3, a critical proapoptotic enzyme that induces DNA breakage. As shown in Figures 2(e) and 2(f), caspase-3 expression was undetectable in macrophages under normal conditions; ox-LDL treatment significantly increased caspase-3 levels in macrophages, and siRNA/Drp1 inhibited this effect. Taken together, these results demonstrated that inhibition of Drp1-related mitochondrial fission significantly reduces ox-LDL-induced macrophage death.

RETRACTED

### 2.3. Inhibition of Drp1-Related Mitochondrial Fission Improves Cholesterol Metabolism in Macrophages

At the molecular level, excessive cholesterol accumulation has been identified as an early inducer of macrophage dysfunction that contributes to the progression of atherosclerosis [32, 33]. Thus, we examined cholesterol metabolism in macrophages transfected with siRNA/Drp1. CD36 and LOX-1 are involved in ox-LDL uptake, while ABCA1 and ABCG1 are involved in cholesterol efflux [34, 35]. A qPCR assay demonstrated that transcription of CD36 and LOX-1 increased significantly in response to ox-LDL (Figures 3(a) and 3(b)). In contrast, transcription of ABCA1 and ABCG1 was markedly reduced after exposure to ox-LDL (Figures 3(c) and 3(d)). Conversely, after transfection of siRNA/Drp1, CD31 and LOX-1 transcription was downregulated and ABCA1 and ABCG1 transcription was upregulated (Figures 3(a)–3(d)). This indicates that inhibition of mitochondrial fission reduces cholesterol uptake and promotes cholesterol efflux. This finding was confirmed through immunofluorescence. As shown in Figures 3(e)–3(g), compared to the control group, CD36 was upregulated and ABCA1 was downregulated after ox-LDL treatment. After transfection of siRNA/Drp1, CD36 expression decreased and ABCA1 expression increased (Figures 3(e)–3(g)). These data confirmed that inhibition of mitochondrial fission improved cholesterol metabolism.

### 2.4. ox-LDL Triggers Oxidative Stress in Macrophages through Drp1-Related Mitochondrial Fission

Oxidative stress and inflammation response are associated with macrophage dysfunction [36–38]. We therefore examined whether mitochondrial fission also regulated oxidative stress in ox-LDL-treated macrophages. Intracellular ROS levels were measured through immunofluorescence. As shown in Figures 4(a) and 4(b), compared to the control group, ox-LDL treatment significantly increased ROS levels, and inhibition of mitochondrial fission inhibited ROS production. We also measured mitochondrial ROS levels. As shown in Figures 4(c) and 4(d), compared to control group, mitochondrial ROS levels increased dramatically after ox-LDL treatment, and this effect was reversed by siRNA/Drp1. Finally, we measured changes in the activity of antioxidative enzymes. As shown in Figures 4(e)–4(g), compared to the control group, GSH, GPX, and SOD activity was significantly downregulated after exposure to ox-LDL. However, inhibition of mitochondrial fission through transfection of siRNA/Drp1 significantly reversed this reduction in GSH, SOD, and GPX activity. Overall, our data illustrated that ox-LDL-induced oxidative stress was attenuated by inhibition of Drp1-related mitochondrial fission.

RETRACTED

### 2.5. ox-LDL Induces Inflammatory Response Dependent on Drp1-Related Mitochondrial Fission in Macrophages

To understand the role of Drp1-related mitochondrial fission in macrophage inflammatory responses, ELISA was used to measure levels of proinflammatory factors in macrophages. As shown in Figures 5(a)–5(d), compared to the control group, ox-LDL upregulated IL-6, IL-12, MCP1, and TNF*α* levels, and siRNA/Drp1 transfection decreased levels of these proinflammatory factors. Consistent with these findings, IL-6, IL-12, MCP1, and TNF*α* transcription was increased by ox-LDL and inhibited by siRNA/Drp1 (Figures 5(e)–5(h)). These data suggest that siRNA/Drp1 attenuated the ox-LDL-induced inflammatory response in macrophages.

### 2.6. ox-LDL Regulates Drp1-Related Mitochondrial Fission through miR-9

We previously reported that miR-9 regulates macrophage function and protects against inflammatory responses through various mechanisms [39]. Subsequent studies further described the strong effects miR-9 exerts on mitochondrial function [40]. We therefore examined whether mitochondrial fission is regulated by miR-9 in ox-LDL-treated macrophages. Indeed, ox-LDL treatment significantly reduced miR-9 levels in macrophages (Figure 6(a)). To determine whether decreased miR-9 is involved in ox-LDL-mediated mitochondrial fission and macrophage dysfunction, cell viability and mitochondrial fission were examined in macrophages cocultured with a miR-9 mimic before ox-LDL treatment. As shown in Figures 6(b)–6(d), compared to the control group, numbers of fragmented mitochondria increased in response to ox-LDL treatment, and the miR-9 mimic inhibited this effect. We also found that transcription of Drp1, but not Fis1, was repressed by miR-9 mimic exposure prior to ox-LDL treatment, suggesting that miR-9 may modulate Drp1 expression at the posttranscriptional level (Figures 6(e) and 6(f)). In addition, a CCK-8 assay demonstrated that the miR-9 mimic maintained macrophage viability after ox-LDL treatment (Figure 6(g)). Similarly, miR-9 mimic restored antioxidative factors to normal levels (Figures 6(h) and 6(i)) and inhibited the transcription of proinflammatory factors (Figures 6(j) and 6(k)) in macrophages. Together, these results highlight the important role of miR-9 in regulating mitochondrial fission, oxidative stress, and inflammatory response in ox-LDL-treated macrophages.

RETRACTED

## 3. Discussion

In this study, we found that ox-LDL treatment activated mitochondrial fission in macrophages. Furthermore, inhibition of mitochondrial fission significantly reduced ox-LDL-mediated macrophage damage. Mechanistically, inhibition of mitochondrial fission increased macrophage viability, repressed oxidative stress, attenuated inflammatory response, and improved cholesterol metabolism. We also found that ox-LDL-induced mitochondrial fission was regulated by miR-9 in macrophages. Reduced miR-9 levels resulted in increased transcription of Drp1, which in turn activated mitochondrial fission. These results define a novel miR-9/Drp1/mitochondrial fission signaling pathway that affects macrophage function and cholesterol metabolism. Treatment strategies targeting miR-9 and mitochondrial fission might therefore benefit patients suffering from AS.

During hyperlipidemia, macrophages play a crucial role in maintaining balanced cholesterol levels by regulating scavenger receptors, cholesterol metabolism enzymes, and cholesterol transporters [22]. After scavenger receptors initially interact with free cholesterol, cholesterol transporters facilitate uptake of free cholesterol by macrophages; mitochondria then use cholesterol to generate ATP through cholesterol metabolism enzymes [41]. Importantly, cholesterol transporters can also facilitate excretion of excess cholesterol from cells [42]. The balance between cholesterol uptake and release therefore affects macrophage function. In this study, we found that genes related to cholesterol uptake were significantly upregulated while the genes related to cholesterol efflux were significantly downregulated in response to ox-LDL, suggesting that hyperlipidemia increases intake and inhibits release of cholesterol in macrophages. Excessive cholesterol accumulation in macrophages promotes foam cell formation during atherogenesis [43]. As far as we know, ours is the first investigation to demonstrate that mitochondrial fission improves cholesterol metabolism in macrophages. However, some topics require further investigation. First, additional studies are required to identify the molecular mechanism underlying mitochondrial fission-mediated normalization of cholesterol receptor levels. In addition, whether decreased mitochondrial fission inhibits mitochondrial cholesterol metabolism in macrophages remains unknown and should be examined.

miRNAs decrease gene expression by binding to the 3′-untranslated region (UTR) of target RNAs, resulting in their degradation [44]. miRNA expression profiles have diagnostic and prognostic value for cancer, and miRNAs may serve as potential targets for antitumor immunotherapies [45]. Several miRNAs that are associated with cholesterol metabolism in macrophages have been identified. For example, miR-144-5p regulates inflammatory response in macrophages by mediating the expression of TLR2 and OLR1 [46]. ox-LDL-induced cholesterol accumulation in macrophages seems to be modulated by miR-33a through the ERK/AMPK/SREBP1 signaling pathway [47]. ox-LDL-induced macrophage apoptosis and oxidative stress are also linked to miR-140-5p [48]. In addition, miR-202-3p upregulation promotes foam cell formation [49]. In this study, we found that miR-9 regulates macrophage cholesterol metabolism. miR-9 exerts important effects on diabetic peripheral neuropathy progression by regulating the OSL1-mediated sonic hedgehog signaling pathway [50]. Macrophage M1 polarization [40], macrophage foam cell formation [51], and macrophage inflammatory response [52] are also regulated by miR-9. More importantly, recent studies have also demonstrated that miR-9 regulates the stabilization of mitochondria-related proteins [31] and mitochondrial tRNA-modifying enzymes [53]. In this study, we identified the regulatory mechanisms underlying miR-9-modified mitochondrial fission in macrophages. However, additional animal studies are needed to confirm our findings.

RETRACTED

In summary, we found that macrophage viability and cholesterol metabolism are regulated by a miR-9/Drp1/mitochondrial fission signaling pathway. miR-9 levels were reduced by ox-LDL treatment, which contributed to upregulation of Drp1 transcription and led to macrophage mitochondrial fission. Excessive mitochondrial fission induced oxidative stress, inflammatory response, and cholesterol metabolism dysregulation in macrophages. These findings suggest that modulating macrophage function via the miR-9/Drp1/mitochondrial fission signaling pathway may be a novel treatment for AS.

## 4. Methods

### 4.1. Cell Culture

Macrophage induction and differentiation from monocytes were performed as previously described [39]. Macrophages were cultured in RPMI 1640 medium (Gibco, NY, USA) supplemented with 10% fetal bovine serum (FBS), penicillin, and streptomycin. ox-LDL at a concentration of 50 *μ*g/mL was also added to the macrophage medium for 24 hours. Additionally, an miR-9 precursor (pre-miR-9) was constructed and transfected into macrophages as previously described [39].

### 4.2. Cell Viability Assay

Macrophage viability was evaluated using a CCK-8 kit (Dojindo, Japan) [54]. Cells were seeded onto 96-well plates at a density of 2.5 × 10^4^ cells/well. Cells were washed twice with PBS and incubated with 100 *μ*L of culture medium containing 10% CCK-8 solution every 12 h after plating at 37°C. Absorbance at 450 nm was quantified using a DTX-880 multimode microplate reader (Beckman, US) [55].

RETRACTED

### 4.3. siRNA Transfection

Macrophages were plated at subconfluence (10^5^ cells in each well of a 6-well plate) without antibiotics, which can interfere with siRNA transfection efficiency. The next day, cells were transfected with Lipofectamine® RNAiMAX transfection reagent (Invitrogen, 13778-150) according to the manufacturer's protocol [56]. Macrophages were transfected with Drp1 siRNA or control siRNA, which were purchased from GenePharma (Shanghai, China), for 24 h. After siRNA transfection, macrophages were serum starved in RPMI 1640 medium for 24 hours prior to the start of the indicated experimental protocols [57]. Assays were performed 48 hours after siRNA transfection.

### 4.4. ELISA Quantification Assay

GSH, SOD, GPX, and proinflammatory factor activity was quantified using Quantikine ELISA Immunoassay kits (R&D Systems). In brief, after macrophages underwent siRNA transfection, 1 mL of fresh cell culture medium was added to each well of a 6-well plate, and conditioned medium was collected 6 hours after elastase exposure [58]. Conditioned media were centrifuged at 3,000 × g for 15 minutes to remove cell debris. Undiluted conditioned media were used to quantify target protein levels according to the manufacturer's instructions [59]. All samples were run in triplicate.

### 4.5. Immunofluorescence

Samples were drop fixed in 10% buffered formalin overnight and cryopreserved in 30% sucrose in PBS overnight [60, 61]. Samples were then blocked with 2% Donkey serum in 0.1% Tween™ 20 in PBS (antibody diluent) for 30 minutes at room temperature. Antibodies were diluted as follows: TOM20 (Abcam, ab186735, 1 : 100), CD36 (Abcam, ab133625, 1 : 200), caspase-3 (Abcam, ab13847, 1 : 250), ABCA1 (Abcam, ab18180, 1 : 200), and incubated at 4°C overnight. Samples were washed three times in PBS and incubated with the proper fluorescent secondary antibody (Alexa Fluor 488/555/647, Invitrogen) diluted 1 : 800 for two hours at room temperature. Samples were washed three times with PBS and incubated with DAPI (Sigma, B2883) for 1 minute. Samples were then washed three times with PBS and mounted with fluoromount (SouthernBiotech) or ProLong™ Gold antifade reagent (Invitrogen, P10144) [62]. Images were taken on a Nikon Eclipse Ti epifluorescence microscope or a Zeiss LSM700 confocal microscope.

### 4.6. Reverse Transcription Real-Time Quantitative PCR

RNA was extracted from cultured cells using the RNeasy mini kit (Qiagen, Germany). cDNA was synthesized using the iScript cDNA Synthesis Kit (Bio-Rad) [63]. Real-time PCR was performed with SYBR Green Master Mix (TOYOBO, Japan) and an ABI 7500 Fast Real-Time PCR System (Applied Biosystems, US). Relative gene expression was determined by normalizing to GAPDH [64].

RETRACTED

### 4.7. ROS Staining

After treatment, cells were washed with cold PBS and then stained with two types of ROS probes [65, 66]. DCFHDA (Molecular Probes, USA) was used to stain intracellular ROS while MitoSOX red mitochondrial superoxide indicator (Molecular Probes, USA) was used to stain mitochondrial ROS [67]. In brief, 5 *μ*g/L DCFHDA and 2 *μ*g/L MitoSOX were added to the medium and incubated for about 30 min in the dark. Cells were then washed three times with PBS and stained with DAPI, and images were taken on a Nikon Eclipse Ti epifluorescence microscope or a Zeiss LSM700 confocal microscope.

### 4.8. Statistics

Results are expressed as mean ± SEM. The Kruskal-Wallis one-way analysis of variance was used to compare each measure when there were three or more independent groups. Comparisons between groups were performed using Dunn's multiple comparisons test when statistically significant differences were identified in ANOVAs. A *p* value < 0.05 was considered significant. The Mann–Whitney test was used to compare two groups. All data were analyzed using Prism 5.0 (GraphPad Software Inc.).

## Figures and Tables

**Figure 1:** ox-LDL activates mitochondrial fission and inhibits mitochondrial fusion in macrophages. (a–c) Immunofluorescence assay of mitochondrial morphology. Average mitochondrial length and ratio of fragmented mitochondria were measured in response to ox-LDL treatment. (d–i) RNA was collected from cells, and Mff, Fis1, Drp1, Mfn1, Mfn2, and Opa1 transcription was measured. ^∗^*p* < 0.05.

**Figure 2:** Inhibition of Drp1-related mitochondrial fission attenuates macrophage death induced by ox-LDL. (a) Cell viability was measured through the CCK-8 assay after ox-LDL and siRNA/Drp1 treatments. (b) LDH release assay was used to detect the concentration of LDH in the medium after ox-LDL and siRNA/Drp1 treatments. (c, d) TUNEL staining was used to analyze apoptosis rates in macrophages in response to LDH and siRNA/Drp1 treatments. (e, f) Caspase-3 expression was detected through immunofluorescence after ox-LDL and siRNA/Drp1 treatment. ^∗^*p* < 0.05.

**Figure 3:** Inhibition of Drp1-related mitochondrial fission improves cholesterol metabolism in macrophages. (a, b) A qPCR assay was used to measure levels of CD36 and LOX-1 after ox-LDL and siRNA/Drp1 treatments. (c, d) ABCA1 and ABCG1 transcription was measured through qPCR after ox-LDL and siRNA/Drp1 treatments. (e–g) Macrophage LOX-1 and ABCA1 levels were measured through immunofluorescence after ox-LDL and siRNA/Drp1 treatments. ^∗^*p* < 0.05.

RETRACTED

**Figure 4:** ox-LDL triggers oxidative stress in macrophages through Drp1-related mitochondrial fission. (a, b) Cellular ROS were measured in an immunofluorescence assay using a DCFHDA probe after ox-LDL and siRNA/Drp1 treatments. (c, d) Mitochondrial ROS were measured in an immunofluorescence assay using a MitoSOX probe after ox-LDL and siRNA/Drp1 treatments. (e–g) Activity of the antioxidative factors GSH, GPX, and SOD was measured through ELISA after ox-LDL and siRNA/Drp1 treatments. ^∗^*p* < 0.05.

**Figure 5:** ox-LDL induces inflammatory response dependent on Drp1-related mitochondrial fission in macrophages. (a–d) A qPCR assay was used to measure IL-6, IL-12, MCP1, and TNF*α* levels in RNA isolated from macrophages after ox-LDL and siRNA/Drp1 treatments. (e–h) ELISA was used to detect IL-6, IL-12, MCP1, and TNF*α* activity in macrophages after ox-LDL and siRNA/Drp1 treatments. ^∗^*p* < 0.05.

**Figure 6:** ox-LDL regulates Drp1-related mitochondrial fission through miR-9. (a) Transcription of miR-9 in response to ox-LDL treatment. (b–d) Mitochondrial morphology was observed using immunofluorescence. (e, f) A qPCR assay was used to measure transcription of Fis1 and Drp1 in macrophages after ox-LDL treatment. (g) Cell viability was measured in a CCK-8 assay after ox-LDL and miR-9 mimic treatments. (h, i) ELISA was used to measure GSH and SOD activity. (j, k) A qPCR assay was used to measure IL-6 and MCP1 levels in macrophages. ^∗^*p* < 0.05.

## Data Availability

All data are contained within the manuscript and additional files.
